The article "Clustering Undergraduate Students Based on Academic Burnout and Satisfaction from the Field Using Partitioning around Medoid" was published in 2023. Journal: Comput Math Methods Med.

# Clustering Undergraduate Students Based on Academic Burnout and Satisfaction from the Field Using Partitioning around Medoid

**DOI:** 10.1155/2023/8898939

**Published:** 2023-05-29

**Authors:** Elaheh Sanjari, Farzaneh Majidian Dehkordi, Hadi Raeisi Shahraki

**Affiliations:** ^1^Student Research Committee, Shahrekord University of Medical Sciences, Shahrekord, Iran; ^2^Department of Epidemiology and Biostatistics, Faculty of Health, Shahrekord University of Medical Sciences, Shahrekord, Iran

## Abstract

**Background:**

Academic satisfaction is known as one of the most important factors in increasing students' efficiency, and academic burnout is one of the most significant challenges of the educational system, reducing student motivation and enthusiasm. Clustering methods try to categorize individuals into a number of homogenous groups.

**Aims:**

To cluster undergraduate students at Shahrekord University of Medical Sciences based on academic burnout and satisfaction with their field of study.

**Materials and Methods:**

The multistage cluster sampling method was used to select 400 undergraduate students from various fields in 2022. The data collection tool included a 15-item academic burnout questionnaire and a 7-item academic satisfaction questionnaire. The average silhouette index was used to estimate the number of optimal clusters. The NbClust package in R 4.2.1 software was used for clustering analysis based on the k-medoid approach.

**Results:**

The mean score of academic satisfaction was 17.70 ± 5.39, while academic burnout averaged 37.90 ± 13.27. The optimal number of clusters was estimated at two based on the average silhouette index. The first cluster included 221 students, and the second cluster included 179 students. Students in the second cluster had higher levels of academic burnout than the first cluster.

**Conclusion:**

It is suggested that university officials take measures to reduce the level of academic burnout through academic burnout training workshops led by consultants to promote the students' interests.

## 1. Introduction

Interest and satisfaction in education are two of the most important effective factors in the development of efficient human resources, and they should be prioritized in educational planning [1]. Satisfaction is a multifactor word that indicates the scientific effectiveness of all educational fields [2]. It is influenced by a variety of personal, social, economic, cultural, and environmental factors [3]. Academic satisfaction is defined as a person's general attitude toward the field of study and how well the desired field meets the person's needs, abilities, desires, and personal characteristics [4]. Students' satisfaction with their field of study is a collection of compatible and incompatible feelings about the field that increase their efficiency and satisfaction [1].

Academic burnout is one of the problems of the educational system at all levels, which causes a waste of human resources and expenses and is related to the student's enthusiasm for education [5]. Academic burnout among students refers to fatigue, having a pessimistic and disinterested sense of homework, and a sense of inadequacy as a student [6]. This means that no matter how much academic burnout there is among students of different levels of education, it especially affects students' academic performance and academic progress, their commitment to educational affairs, their low academic participation during and after education, and their motivation and enthusiasm towards education [5, 7, 8]. Neumann believes that burnout is one of the most important research topics in universities. He believes that there are various reasons for examining the issue of burnout, the most important of which are (a) academic burnout affects the relationship of students with the university and faculty; (b) academic burnout can reduce the interest and enthusiasm of students to continue their studies; and (c) academic burnout can be an important and essential tool for understanding various actions such as academic performance during education [5].

The topic of satisfaction with the field of study is a variable that has a close relationship with academic burnout at the individual level and from the perspective of social psychology. Moore and Loosemore discovered a link between academic burnout and overall course satisfaction [9]. Previous research has found that factors related to the field of study, such as satisfaction with the field of study, affect academic burnout [10]. Therefore, it is necessary to identify the factors that are related to academic burnout and consider the importance of academic burnout and satisfaction with the field of study.

This study tries to extend previous studies in this field in several ways. First, we use the clustering method which is a multivariate analysis considering the simultaneous modeling of academic burnout and satisfaction with the field of study. Second, although the traditional clustering approaches are more popular, they suffer from the initial assignment of individuals and outliers. In this study, the method of partitioning around medoid was implemented which is a robust technique without any limitations. Third, this study helps motivate researchers to implement modern statistical analysis, which leads to more insightful findings. Due to the lack of related studies, this study was conducted with the aim of clustering students based on academic burnout and satisfaction with the field of study.

## 2. Materials and Methods

The current study is a cross-sectional type, and its statistical population includes all students of Shahrekord University of Medical Sciences (SKUMS), Shahrekord, Iran, in the 2022 year. A multistage cluster sampling method was implemented, and from the list of faculties in SKUMS, three faculties were randomly selected. In the next stage, from each faculty, three departments were selected at random. Finally, by referring to several classes for each of the selected departments, the questionnaires were distributed among the students who were willing to participate in the study.

According to the study of Anbari et al., and taking into account the correlation of 0.15 as well as taking into account the first and second types of errors equal to 0.05 and 0.20, the minimum required sample size was estimated at 350 students, which considering the dropout rate of 13%, means 400 students were included in the study [11].

The academic burnout questionnaire was extracted from the Maslach or Mezlach academic burnout scale by Rostami et al. [12]. This questionnaire has 15 questions that include 7 options that are never = 0, very rarely = 1, relatively little = 2, sometimes = 3, relatively much = 4, most of the time = 5, and always = 6. The scoring method for questions 11 to 15 is reversed. The validity and reliability of the Persian version of this questionnaire have already been confirmed [13, 14].

The academic satisfaction questionnaire created by Lent et al. [15] measures the satisfaction of students both in general and in aspects of their educational experiences. This questionnaire contains 7 items with a 5-point Likert scale as follows: Completely agree = 5, Agree = 4, Have no opinion = 3, Disagree = 2, and Completely disagree = 1). The score range of this questionnaire will be between 7 and 35, and the higher the score obtained from this questionnaire, the higher the level of academic satisfaction. Lent et al. have reported the reliability of this scale using internal consistency of 0.86 and 0.87, and its validity has been confirmed through correlation with academic resistance, life satisfaction, and other cognitive-social variables [15]. In Hashemi et al.'s research, Cronbach's alpha and Spearman-Brown classification were used to determine the reliability of this scale which were 0.82 and 0.77, respectively [16].

## 3. Statistical Methods

Mean ± SD and frequency (%) were used to report descriptive statistics for quantitative and qualitative variables, respectively. To report correlations between quantitative variables, Pearson's correlation was used, and the association between qualitative variables was investigated using the Chi-square test or Fisher's exact test. Also, an independent T-test and one-way analysis of variance were used to compare numerical values in two or more independent groups, respectively.

Partitioning around medoid (PAM) clustering was proposed in 1990 by Kaufman and Rousseuw. The medoid of each cluster is the observation of the same cluster that is most similar to its other members. In this method, the dissimilarity of two observations is calculated and then shown in the form of a dissimilarity matrix [17, 18].

The algorithm of the PAM method is as follows:

1. Determining the number of clusters (*k*)
2. Select *k* observation to become the medoids
3. Calculation of the dissimilarity matrix based on the academic burnout and satisfaction scores
4. Allocating each student into the cluster which had the lowest dissimilarity with the medoids
5. Updating each cluster
6. Recalculation of the dissimilarity matrix

If each observation has the least dissimilarity with its cluster representative, the algorithm terminates; otherwise, return to step 4. Compared to *k*-means clustering, *k*-medoid clustering is less sensitive to outliers and is applicable even for qualitative variables. To determine the number of optimal clusters, the NbClust package in the R 3.5.3 software was used. In this package, statistical indicators are used to determine the number of optimal clusters. An efficient method to determine the number of optimal clusters is the average silhouette method [17, 18].

This method measures the clustering quality of each cluster and determines how well each observation is in its own cluster. The range of this method is between -1 and 1, and the higher values indicate better clustering quality [18].

## 4. Ethical Considerations

In the questionnaires, the names and other personal characteristics of the participating students will not be asked, and all information will be analyzed collectively. Also, the purpose of the research will be explained to the students before the questionnaires are administered. This research project was approved by the Ethics Committee of SKUMS (Ethics code: IR.SKUMS.REC.1398.042).

## 5. Results

Out of 400 students participating in this study, 213 (53.2%) were between the ages of 21 and 23, 303 (75.8%) were female, and 351 (87.8%) were single. Also, the majority of students had Fars ethnicity (52.3%) and lived in dormitories (71.5%). The overall mean ± SD of academic satisfaction was 17.70 ± 5.39 with a minimum of 7 and a maximum of 35. Single students with a mean score of 17.91 ± 5.26 had a significantly higher level of academic satisfaction compared to married students with a mean score of 16.14 ± 6.07 (*P* = 0.03). Moreover, the mean ± SD of satisfaction in environmental health engineering students was 21.30 ± 6.57, significantly higher than the students of other fields (*P* < 0.001) (Table 1).

The overall mean ± SD of academic burnout was 37.90 ± 13.26 with a minimum of 4 and a maximum of 78. The mean score of academic burnout among the students between 21 and 23 years old was significantly higher than the younger students (39.56 ± 11.19 versus 35.43 ± 15.52, *P* = 0.02). Academic burnout was at the highest level for the students of environmental health engineering with 42.20 ± 11.94. This level of academic burnout was significantly higher than the mean score of burnout among the public health (33.60 ± 13.62) and midwifery (31.33 ± 15.03) students (Table 1).

The associations between wealth-related factors with satisfaction and academic burnout were summarized in Table 2. The level of satisfaction was significantly lower among the students with higher levels of self-income (*P* = 0.03) and family income (*P* = 0.002), but no significant difference was found between self-income (*P* = 0.14) and family income (*P* = 0.89) with academic burnout (Table 2).

By using the NbClust package, the optimal number of clusters was estimated to be two, so 221 students were categorized in the first cluster and 179 students in the second cluster.  Table 3 is devoted to investigating associations between demographic variables and suggested clusters. Although we did not find any significant association, the percentage of younger students (34.1% versus 30.8%), females (77.1% versus 74.7%), public health students (19.6% versus 12.2%), and midwifery students (14.5% versus 10.0%) was higher in the second cluster. Besides, the percentage of students who had their own car (9.0% versus 11.7%) and self-income (12.7% versus 12.8%) was lower in the first cluster without any statistical significance (Table 4).

Based on the PAM clustering method, the undergraduate students were divided into two groups based on satisfaction and burnout. The scatter plot of the suggested clusters based on satisfaction and academic burnout is displayed in Figure 1.

As was shown, students in the first cluster had higher levels of satisfaction and academic burnout compared to the second cluster.

## 6. Discussion

The purpose of this study was to group undergraduate students at Shahrekord University of Medical Sciences based on academic burnout and satisfaction with their field of study. This study found that male students had a higher average academic burnout than female students, but there was no significant difference in burnout between the sexes, which was consistent with previous research. The average academic burnout was higher in male students than female students without any statistically significant in the study by Yu and Chae. They stated that when male students experience academic burnout, they distance themselves from their studies more than female students, resulting an earlier dropout [19]. Shokrpour et al., on the other hand, conducted a study to identify the most important determinants of academic burnout among medical students. This study found a significant difference between the academic burnout of males and females, which contradicts the findings of this study. It may be due to the different range of ages or gender proportions of the participants in these studies [20].

Our findings revealed that single students had a higher level of academic burnout, despite the fact that the observed difference was not statistically significant. In this regard, Rahmatpour et al. showed that married students have lower academic burnout grades than single students. One reason is that married students have a more purposeful life, better time management, and more motivation to continue and finish their studies [21]. Another significant finding of this study was a significant and negative correlation between academic burnout and academic satisfaction. In this regard, Kim and Lee justified that students who are dissatisfied with their university life have high academic burnout. It appears that interest in the field of study is important in reducing academic burnout [22]. Abuddous et al. showed negative and significant correlations between the dimensions of burnout and satisfaction. This finding can be justified by stating that the emotional state of second-year students is still premature in terms of satisfaction with the field of study. The authors claimed that junior and senior students consistently expressed their level of satisfaction with their field of study [23].

Adib et al. showed that there is a negative and significant correlation between academic burnout and academic satisfaction. Students who are uninterested and unmotivated may not try hard enough, and this inattention and lack of effort will lead to academic burnout. Therefore, by reducing the factors that cause academic burnout, such as increasing the motivation and interest in the course and field of study in students, the satisfaction of the field of study can be improved [24].

In this study, academic satisfaction among nondormitory students was higher than among dormitory students. However, the observed differences were not statistically significant. In this regard, in the study of Kamalpour et al., it was shown that students who live with their families had better academic satisfaction compared to students who live in dormitories. The reason for this difference can be attributed to the atmosphere prevailing in these environments [25]. Also, students who live in the dormitory experience pressures such as being away from their families, as well as the stress of the student period and the decrease in academic motivation, which causes this group of students to have less academic satisfaction [26]. Besides, in the study of Taheri et al., it was shown that there was a significant association between academic majors and academic burnout. They stated that factors such as the nature of the field of study, the number and difficulty of the courses offered during the study, work pressure, and issues related to the future career lead to academic burnout [27].

Unfortunately, we found no previous studies on clustering students based on academic burnout and satisfaction to compare their related findings, which was the main limitation of this study. Also, it was better to ask about the state of love instead of marital status which is an important factor affecting the psychological state of contemporary college students. Finally, conducting a multicenter study with a larger sample size and considering other potential confounding factors that can be generalized to the Iranian student population is highly suggested. In addition, to consider more economic factors, more diverse and reliable economic variables should be considered. For future investigation, clustering students based on academic burnout, depression, anxiety, and stress is highly suggested.

## 7. Conclusion

Given that the university's main mission is to train the specialized manpower required by society and to lay the groundwork for the country's development, and given that medical education is of particular importance due to the graduates' responsibility for human lives, efforts should be made to improve the quality of medical education. Such studies help identify a group of students with higher levels of academic burnout and required more attention. It is suggested that university officials take measures to reduce the level of academic burnout through academic burnout training workshops led by consultants, particularly at the start of the first academic semester, in order to promote the students' interests.

## Figures and Tables

**Figure 1:** scatter plot of the suggested clusters based on satisfaction and academic burnout.

**Table 1:** The comparison of satisfaction and academic burnout in different categories of demographic variables.

Variable	Subgroup	Satisfaction	*P* value	Academic burnout	*P* value
Age	≤20 years (*n* = 129)	17.53 ± 5.08	0.13	35.43 ± 15.52	**0.02**
	21-23 years (*n* = 213)	18.12 ± 5.73		39.56 ± 11.19	
	≥24 years (*n* = 58)	16.53 ± 4.60		37.28 ± 14.16	

Gender	Female (*n* = 303)	17.89 ± 5.62	0.21	37.82 ± 13.68	0.83
	Male (*n* = 97)	17.10 ± 4.55		38.15 ± 11.93	

Marital status	Single (*n* = 351)	17.91 ± 5.26	**0.03**	38.24 ± 13.01	0.17
	Married (*n* = 49)	16.14 ± 6.07		35.47 ± 14.88	

Ethnicity	Lor (*n* = 147)	18.05 ± 5.66	0.37	39.32 ± 12.49	0.21
	Fars (*n* = 210)	17.65 ± 5.37		36.82 ± 13.73	
	Other (*n* = 43)	16.74 ± 4.47		38.30 ± 13.34	

Dormitory residence	No (*n* = 114)	18.13 ± 6.30	0.31	39.15 ± 14.44	0.23
	Yes (*n* = 286)	17.52 ± 4.98		37.40 ± 12.76	

Major	Public health (*n* = 61)	17.26 ± 5.61	**<0.001**	33.60 ± 13.62	**<0.001**
	Environmental health (*n* = 62)	21.30 ± 6.57		42.20 ± 13.45	
	Laboratory sciences (*n* = 48)	16.50 ± 3.95		38.38 ± 11.94	
	Nursing (*n* = 63)	16.79 ± 3.72		39.89 ± 11.08	
	Radiologic technology (*n* = 25)	17.28 ± 5.06		37.68 ± 14.01	
	Anesthesia (*n* = 46)	15.78 ± 3.76		39.22 ± 13.02	
	Surgical technology (*n* = 47)	19.15 ± 5.86		40.36 ± 11.22	
	Midwifery (*n* = 48)	16.71 ± 5.49		31.33 ± 15.03	

^∗^ *P* < 0.05 is considered statistically significant.

**Table 2:** The comparison of satisfaction and academic burnout in different categories of wealth-related variables.

Variable	Subgroup	Satisfaction	*P* value	Academic burnout	*P* value
Own car	No (*n* = 359)	17.86 ± 5.20		38.20 ± 12.96	0.17
	Yes (*n* = 41)	16.29 ± 6.70		35.22 ± 15.58	

Own laptop	No (*n* = 265)	17.66 ± 5.66	0.83	37.76 ± 13.60	0.77
	Yes (*n* = 135)	17.78 ± 5.24		38.17 ± 12.61	

Self-income	Nothing (*n* = 349)	17.93 ± 5.30	**0.03**	38.10 ± 13.01	0.14
	<50$ per months (*n* = 23)	17.74 ± 6.23		37.61 ± 15.27	
	50 to 100$ per months (*n* = 13)	14.92 ± 5.02		41.31 ± 14.59	
	>100$ per months (*n* = 15)	14.73 ± 5.02		30.67 ± 13.79	

Family income	<200$ per months (*n* = 101)	19.44 ± 6.23	**0.002**	38.02 ± 14.05	0.89
	200 to 400$ per months (*n* = 192)	17.05 ± 4.74		37.42 ± 12.63	
	400 to 600$ per months (*n* = 87)	17.16 ± 5.06		38.71 ± 13.17	
	>600$ per months (*n* = 20)	17.45 ± 6.41		38.35 ± 16.07	

^∗^ *P* < 0.05 is considered statistically significant.

**Table 3:** The association between demographic variables and suggested clusters.

Variable	Subgroup	Cluster number 1	Cluster number 2	*P* value
Age	≤20 years (*n* = 129)	68 (30.8)	61 (34.1)	0.61
	21-23 years (*n* = 213)	118 (53.4)	95 (53.1)	
	≥24 years (*n* = 58)	35 (15.8)	23 (12.8)	

Gender	Female (*n* = 303)	165 (74.7)	138 (77.1)	0.64
	Male (*n* = 97)	56 (25.3)	41 (22.9)	

Marital status	Single (*n* = 351)	199 (90.0)	152 (84.9)	0.13
	Married (*n* = 49)	22 (10.0)	27 (15.1)	

Ethnicity	Lor (*n* = 147)	85 (38.5)	62 (34.6)	0.69
	Fars (*n* = 210)	114 (51.6)	96 (53.6)	
	Other (*n* = 43)	22 (10.0)	21 (11.7)	

Dormitory residence	No (*n* = 114)	69 (31.2)	45 (25.1)	0.18
	Yes (*n* = 286)	152 (68.8)	134 (74.9)	

Major	Public health (*n* = 62)	27 (12.2)	35 (19.6)	0.14
	Environmental health (*n* = 61)	41 (18.6)	20 (11.2)	
	Laboratory sciences (*n* = 48)	26 (11.8)	22 (12.3)	
	Nursing (*n* = 63)	35 (15.8)	28 (15.6)	
	Radiologic technology (*n* = 25)	13 (5.9)	12 (6.7)	
	Anesthesia (*n* = 46)	26 (11.8)	20 (11.2)	
	Surgical technology (*n* = 47)	31 (14.0)	16 (8.9)	
	Midwifery (*n* = 48)	22 (10.0)	26 (14.5)	

^∗^ *P* < 0.05 is considered statistically significant.

**Table 4:** the association between wealth related variables and suggested clusters.

Variable	Subgroup	Cluster number 1	Cluster number 2	*P* value
Own car	No (*n* = 359)	201 (91.0)	158 (88.3)	0.41
	Yes (*n* = 41)	20 (9.0)	21 (11.7)	

Own laptop	No (*n* = 265)	141 (63.8)	124 (69.3)	0.29
	Yes (*n* = 135)	80 (36.2)	55 (30.7)	

Self-income	Nothing (*n* = 349)	193 (87.3)	156 (87.2)	0.52
	< 50$ per months (*n* = 23)	15 (6.8)	8 (4.5)	
	50 to 100$ per months (*n* = 13)	7 (3.2)	6 (3.4)	
	> 100$ per months (*n* = 15)	6 (2.7)	9 (5.0)	

Family income	< 200$ per months (*n* = 101)	54 (24.4)	47 (26.3)	0.95
	200 to 400$ per months (*n* = 192)	107 (48.4)	85 (47.5)	
	400 to 600$ per months (*n* = 87)	48 (21.7)	39 (21.8)	
	> 600$ per months (*n* = 20)	12 (5.4)	8 (4.5)	

^∗^ *P* < 0.05 is considered statistically significant.

## Data Availability

The data used to support the findings of this study are available from the corresponding author upon request.
